RETRACTED

# TNF-α Induces Cytosolic Phospholipase A_2_ Expression in Human Lung Epithelial Cells via JNK1/2- and p38 MAPK-Dependent AP-1 Activation

**DOI:** 10.1371/journal.pone.0072783

**Published:** 2013-09-19

**Authors:** I-Ta Lee, Chih-Chung Lin, Shin-Ei Cheng, Li-Der Hsiao, Yu-Chun Hsiao, Chuen-Mao Yang

**Affiliations:** 1 Department of Anesthetics, Chang Gung Memorial Hospital at Lin-Kou and College of Medicine, Chang Gung University, Kwei-San, Tao-Yuan, Taiwan; 2 Department of Physiology and Pharmacology and Health Aging Research Center, College of Medicine, Chang Gung University, Kwei-San, Tao-Yuan, Taiwan; Department of Immunology, China

## Abstract

**Background:**

Cytosolic phospholipase A_2_ (cPLA_2_) plays a pivotal role in mediating agonist-induced arachidonic acid (AA) release for prostaglandin (PG) synthesis during inflammation triggered by tumor necrosis factor-α (TNF-α). However, the mechanisms underlying TNF-α-induced cPLA_2_ expression in human lung epithelial cells (HPAEpiCs) were not completely understood.

**Principal Findings:**

We demonstrated that TNF-α induced cPLA_2_ mRNA and protein expression, promoter activity, and PGE_2_ secretion in HPAEpiCs. These responses induced by TNF-α were inhibited by pretreatment with the inhibitor of MEK1/2 (PD98059), p38 MAPK (SB202190), JNK1/2 (SP600125), or AP-1 (Tanshinone IIA) and transfection with siRNA of TNFR1, p42, p38, JNK2, c-Jun, c-Fos, or ATF2. We showed that TNF-α markedly stimulated p42/p44 MAPK, p38 MAPK, and JNK1/2 phosphorylation which were attenuated by their respective inhibitors. In addition, TNF-α also stimulated c-Jun and ATF2 phosphorylation which were inhibited by pretreatment with SP600125 and SB202190, respectively, but not PD98059. Furthermore, TNF-α-induced cPLA_2_ promoter activity was abrogated by transfection with the point-mutated AP-1 cPLA_2_ construct. Finally, we showed that TNF-α time-dependently induced p300/c-Fos/c-Jun/ATF2 complex formation in HPAEpiCs. On the other hand, TNF-α induced *in vivo* binding of c-Jun, c-Fos, ATF2, and p300 to the cPLA_2_ promoter in these cells. In an *in vivo* study, we found that TNF-α induced leukocyte count in BAL fluid of mice and cPLA_2_ mRNA levels in lung tissues via MAPKs and AP-1.

**Significance:**

Taken together, these results demonstrated that TNF-α-induced cPLA_2_ expression was mediated through p38 MAPK- and JNK1/2-dependent p300/c-Fos/c-Jun/ATF2 complex formation in HPAEpiCs.

## Introduction

Lung inflammation is a pivotal event in the pathogenesis of chronic obstructive pulmonary disease (COPD) and asthma [1]. Several lipid mediators, such as eicosanoids generated from arachidonic acid (AA) have been identified in situ in airway secretion of asthmatics [2], [3]. The generation of eicosanoids is first initiated through the release of AA from membrane phospholipids hydrolyzed by the action of phospholipase A_2_ (PLA_2_) enzymes [4]. AA is further converted to prostaglandins (PGs), such as PGE_2_ by the constitutive enzyme cyclooxygenase (COX)-1 or the inducible COX-2 in various cell types [5], [6]. The PLA_2_ superfamily is composed of three main types of lipolytic enzymes, including secretory PLA_2_, the 85 kDa cytosolic group IV PLA_2_ (cPLA_2_), and a calcium-independent group VI PLA_2_ in mammalian cells [7]. cPLA_2_ is the only one that plays a key role in mediating agonist-induced AA release for eicosanoid production in various cell types [8]. It has been demonstrated that activation of the MAPKs, including p42/p44 MAPK, p38 MAPK, and JNK1/2, by pro-inflammatory stimuli leads to the phosphorylation of cPLA_2_ at Ser^505^ and Ser^727^ [9] with Ca^2+^/calmodulin kinase II-dependent phosphorylation of Ser^515^ associated with increased enzymatic activity [10]. cPLA_2_ has been shown to be implicated in acute lung injury induced by sepsis [11] and bronchial reactivity associated with anaphylaxis [12]. Furthermore, increased PGE_2_ synthesis is dependent on an increase in cPLA_2_ activity in various cell types [13], [14]. Elevated levels of pro-inflammatory cytokines, including TNF-α in the bronchoalveolar lavage fluid have been detected in allergic asthmatic patients. TNF-α exerts as a potent stimulus in inflammatory responses through up-regulation of target genes, such as cPLA_2_ in various cell types [15], [16]. The expression of cPLA_2_ induced by TNF-α may be integrated to the signaling networks that augment lung inflammation by enhancing PGE_2_ synthesis. Although cPLA_2_ has been shown to mediate inflammatory reactions, the detail mechanisms underlying TNF-α-induced cPLA_2_ expression and PGE_2_ synthesis in human lung epithelial cells (HPAEpiCs) were not completely understood.

RETRACTED

Several extracellular stimuli elicit a broad spectrum of biological responses through activation of MAPK cascades leading to phosphorylation of specific target proteins [17]. Moreover, we have demonstrated that TNF-α causes a rapid phosphorylation of p42/p44 MAPK or p38 MAPK and up-regulation of COX-2 in human airway smooth muscle cells [18]. In addition, JNK1/2, p42/p44 MAPK, and p38 MAPK have also been shown to be involved in lipopolysaccharide (LPS)-induced cPLA_2_ induction in canine tracheal smooth muscle cells [19]. On the other hand, we have also indicated that MAPKs and NF-κB were involved in TNF-α-induced PGE_2_ release in human airway smooth muscle cells [20]. Therefore, in this study, we investigated the roles of MAPKs in TNF-α-mediated cPLA_2_ expression and PGE_2_ synthesis in HPAEpiCs.

AP-1 is a heterogeneous collection of dimeric transcription factors comprising Jun, Fos, and ATF subunits. Among AP-1 subunits, c-Jun is the most important transcriptional activator in inflammatory status [21]. AP-1 activity is regulated by multiple mechanisms, including phosphorylation by various MAPKs [22]. Among MAPKs, JNK1/2 predominantly plays an important role in TNF-α-induced AP-1 activity, which contributes to the induction of TNF-α-targeted genes [23]. Histone acetyltransferases (HATs), such as p300 and CREB-binding protein functioning as transcriptional co-activators and signal integrators have been proved to play a vital role in expression of inflammatory genes, such as cPLA_2_ or COX-2 [20], [24]. By this model, the activities of HATs must be tightly regulated in response to various stimuli, such as TNF-α, IL-1β, and bacterial toxins [25], [26]. It has been demonstrated that pulmonary inflammation, exacerbated asthma, and COPD induced by exposure to diesel exhaust particulate matter are related to the p300 activation and recruitment to the promoter region of COX-2 [27]. Thus, the role of p300 in TNF-α-mediated AP-1 activation leading to cPLA_2_ expression was also investigated in HPAEpiCs.

In addressing these questions, experiments were performed to investigate the mechanisms underlying TNF-α-induced cPLA_2_ expression and PGE_2_ synthesis in HPAEpiCs. These findings suggested that in HPAEpiCs, TNF-α-induced cPLA_2_ expression associated with PGE_2_ release was, at least in part, mediated through JNK1/2- and p38 MAPK-dependent p300-AP-1 signaling pathway. These results demonstrated that MAPKs and AP-1 may be the critical components implicated in cPLA_2_ expression and PGE_2_ synthesis in TNF-α-challenged HPAEpiCs.

## Methods

### Materials

Recombinant human TNF-α was from R&D System (Minneapolis, MN). Anti-cPLA_2_, anti-GAPDH, anti-TNFR1, anti-p42, anti-p38, anti-JNK2, anti-c-Jun, anti-c-Fos, anti-ATF2, and anti-p300 antibodies were from Santa Cruz (Santa Cruz, CA). Anti-phospho-p42/p44 MAPK, anti-phospho-p38 MAPK, anti-phospho-JNK1/2, anti-phospho-ATF2, and anti-phospho-c-Jun antibodies were from Cell Signaling (Danver, MA). Actinomycin D (Act. D), cycloheximide (CHI), SP600125, PD98059, SB202190, AACOCF_3_, and Tanshinone IIA were from Biomol (Plymouth Meeting, PA). AH 6809, SC-19220, and GW627368X were from Cayman (Ann Arbor, MI). Other chemicals were from Sigma (St. Louis, MO).

### Cell culture

Human pulmonary alveolar epithelial cells (HPAEpiCs, type II alveolar epithelial cells) were purchased from the ScienCell Research Lab. (San Diego, CA) and grown as previously described [28].

RETRACTED

### Western blot analysis

Growth-arrested HPAEpiCs were incubated with thrombin at 37°C for the indicated time intervals. The cells were washed, scraped, collected, and centrifuged at 45000× *g* at 4°C for 1 h to yield the whole cell extract, as previously described [28]. Samples were denatured, subjected to SDS-PAGE using a 10% running gel, transferred to nitrocellulose membrane, incubated with an anti-cPLA_2_ antibody for 24 h, and then incubated with an anti-mouse horseradish peroxidase antibody for 1 h. The immunoreactive bands were detected by ECL reagents.

### Real-time PCR

Total RNA was extracted using TRIzol reagent. mRNA was reverse-transcribed into cDNA and analyzed by real-time RT-PCR. Real-time PCR was performed using SYBR Green PCR reagents (Applied Biosystems, Branchburg, NJ) and primers specific for cPLA_2_ and GAPDH mRNAs. The levels of cPLA_2_ expression were determined by normalizing to GAPDH expression.

### Measurement of cPLA_2_ luciferase activity

For construction of the cPLA_2_-luc plasmid, human cPLA_2_ promoter, a region spanning −2375 to +75 bp, was cloned into pGL3-basic vector (Promega, Madison, WI). cPLA_2_-luc activity was determined as previously described [28] using a luciferase assay system (Promega, Madison, WI). Firefly luciferase activities were standardized for β-gal activity.

### Measurement of PGE_2_ generation

Cells were cultured in 6-well culture plates. After reaching confluence, cells were treated with TNF-α for the indicated times. After treatment, the medium were collected and stored at −80°C until being assayed. PGE_2_ was assayed using the PGE_2_ enzyme immunoassay kit (Cayman) according to the manufacturer's instructions.

### Transient transfection with siRNAs

Human siRNAs of scrambled, TNFR1, p42, p38, JNK2, c-Jun, c-Fos, and ATF2 were from Sigma (St. Louis, MO). Transient transfection of siRNAs (100 nM) was performed using a Lipofectamine™ RNAiMAX reagent according to the manufacturer's instructions.

### Chromatin immunoprecipitation assay

To detect the association of nuclear proteins with human cPLA_2_ promoter, chromatin immunoprecipitation (ChIP) analysis was conducted as previously described [20]. DNA immunoprecipitated using an anti-p300, anti-ATF2, anti-c-Fos, or anti-c-Jun antibody was purified. The DNA pellet was re-suspended in H_2_O and subjected to PCR amplification with the forward primer 5′-GAATTCAACCTGATTTCATTTTCTTCC-3′ and the reverse primer 5′-CTTCAGGCTCCTCAATGCCTCTAGCTTTCAG-3′, which were specifically designed from the cPLA_2_ promoter region. PCR products were analyzed on ethidium bromide-stained agarose gels (1%).

RETRACTED

### Co-immunoprecipitation assay

Cell lysates containing 1 mg of protein were incubated with 2 µg of an anti-p300 antibody at 4°C for 24 h, and then 10 µl of 50% protein A-agarose beads was added and mixed for 24 h at 4°C. The immunoprecipitates were collected and washed three times with a lysis buffer without Triton X-100. 5X Laemmli buffer was added and subjected to electrophoresis on SDS-PAGE, and then blotted using an anti-c-Fos, anti-c-Jun, anti-ATF2, or anti-p300 antibody.

### Animal care, ethics statement, and experimental procedures

Male ICR mice aged 6–8 weeks were purchased from the National Laboratory Animal Centre (Taipei, Taiwan) and handled according to the guidelines of Animal Care Committee of Chang Gung University approved for this study (IACUC approval number: 12-048) and National Institutes of Health Guides for the Care and Use of Laboratory Animals. All treatments were performed under pentobarbital sodium anesthesia, and all efforts were made to minimize suffering. ICR mice were anesthetized with intraperieritoneal injection of 200 µl of pentobarbital sodium (5 mg/ml) and placed individually on a board in a near vertical position and the tongues were withdrawn with a lined forceps. TNF-α (0.125 mg/kg body weight) was placed posterior in the throat and aspirated into lungs. Control mice were administrated sterile 0.1% BSA. Mice regained consciousness after 15 min. Mice were i.p. given one dose of PD98059, SB202190, SP600125, Tanshinone IIA, AH 6809, SC-19220, GW627368X, or AACOCF_3_ (2 mg/kg) for 1 h prior to TNF-α treatment, and sacrificed after 24 h.

### Isolation of bronchoalveolar lavage (BAL) fluid

Mice were injected with TNF-α at a dose of 0.75 mg/kg and sacrificed 24 h later. BAL fluid was performed through a tracheal cannula using 1 ml aliquots of ice-cold PBS medium. BAL fluid was centrifuged at 500× *g* at 4°C, and cell pellets were washed and re-suspended in PBS. Leukocyte count was determined by a hemocytometer.

### Analysis of data

All data were estimated and made using a GraphPad Prism Program (GraphPad, San Diego, CA, USA). Data were expressed as the mean±S.E.M. and analyzed by one-way ANOVA followed with Tukey's post-hoc test. *P*<0.05 was considered significant.

## Results

### TNF-α induces cPLA_2_ expression and PGE_2_ release in HPAEpiCs

To determine the effect of TNF-α on cPLA_2_ expression, cells were incubated with TNF-α for the indicated time intervals. As shown in Fig. 1A, TNF-α induced cPLA_2_ protein expression in a time-dependent manner with a maximal response within 16–24 h. Moreover, TNF-α also enhanced cPLA_2_ mRNA accumulation in a time-dependent manner with a maximal response within 4–6 h (Fig. 1B). On the other hand, TNF-α markedly induced cPLA_2_ promoter activity in these cells (Fig. 1B). cPLA_2_ is the major form of PLA_2_, which selectively hydrolyzes membrane phospholipids at the sn-2 position and is the rate-limiting enzyme in the release of AA [20]. AA is further converted to PGs (i.e. PGE_2_) by the constitutive enzyme COX-1 or by the inducible COX-2. In our previous study, up-regulation of COX-2 has been shown to induce PGE_2_ synthesis by TNF-α [18]. Therefore, the synthesis of PGE_2_ is a good index of AA release that is more sensitive than [^3^H]AA mobilization [18]. We further tested the effect of TNF-α on PGE_2_ synthesis as a parameter of cPLA_2_ activity. As shown in Fig. 1C, TNF-α induced a time-dependent increase in PGE_2_ synthesis. These results suggested that TNF-α induces cPLA_2_ expression associated with PGE_2_ generation in HPAEpiCs.

RETRACTED

**Figure 1:** TNF-α induces cPLA_2_ protein and mRNA expression. Cells were incubated with TNF-α for the indicated time intervals. (A) The protein levels of cPLA_2_ were determined by Western blot, (B) the mRNA levels of cPLA_2_ were determined by real-time PCR, and the promoter activity of cPLA_2_ was determined in the cell lysates. (C) Cells were incubated with TNF-α (30 ng/ml) for the indicated time intervals. The media were collected and analyzed for PGE_2_ release. Data are expressed as mean±S.E.M. of three independent experiments. *P<0.05; ^#^ *P*<0.01, as compared with the cells exposed to vehicle alone.

### TNF-α induces cPLA_2_ expression via TNFR1 in HPAEpiCs

To further determine whether TNF-α-induced cPLA_2_ expression required transcription or translation, cells were stimulated with TNF-α (30 ng/ml) in the presence of an inhibitor of transcriptional level, actinomycin D (Act. D) or translational level, cycloheximide (CHI) and cPLA_2_ protein expression was determined by Western blot. As shown in Figs. 2A and B, TNF-α-mediated cPLA_2_ protein expression and PGE_2_ release was abolished by either Act. D or CHI in a concentration-dependent manner, while cPLA_2_ mRNA levels were only attenuated by Act. D. Taken together, these findings demonstrated that the induction of cPLA_2_ expression by TNF-α depends on *de novo* protein synthesis in HPAEpiCs. Most of TNF-α actions are elicited through TNFR1 [29]. Thus, we investigated whether TNF-α induced cPLA_2_ expression via TNFR1 in these cells. As shown in Fig. 2C, transfection with TNFR1 siRNA markedly reduced TNFR1 protein expression, and then inhibited TNF-α-induced cPLA_2_ expression in HPAEpiCs. Therefore, TNFR1 mainly plays a key role in TNF-α-induced inflammatory responses.

**Figure 2:** TNF-α induces cPLA_2_ expression via TNFR1 in HPAEpiCs. (A) Cells were pretreated with Act. D or CHI for 1 h, and then incubated with TNF-α for 24 h. The protein levels of cPLA_2_ were determined by Western blot. (B) Cells were pretreated with Act. D (1 µM) or CHI (1 µM) for 1 h, and then incubated with TNF-α for 6 h (for cPLA_2_ mRNA levels) or 24 h (for PGE_2_ release). cPLA_2_ mRNA levels were determined by real-time PCR. The media were collected and analyzed for PGE_2_ release. (C) Cells were transfected with scrambled or TNFR1 siRNA, and then incubated with TNF-α for 24 h. The protein expression of TNFR1 and cPLA_2_ were determined. Data are expressed as mean±S.E.M. of three independent experiments. ^#^ *P*<0.01, as compared with the cells exposed to TNF-α alone.

RETRACTED

### p42/p44 MAPK is involved in TNF-α-induced cPLA_2_ expression in HPAEpiCs

Previous studies demonstrated that TNF-α could induce MAPKs activation in human airway smooth muscle cells [18], [20]. Thus, we further investigated whether TNF-α-induced cPLA_2_ expression was also mediated via p42/p44 MAPK in HPAEpiCs. As shown in Figs. 3A and B, pretreatment with PD98059 (an inhibitor of MEK1/2) attenuated TNF-α-induced cPLA_2_ protein and mRNA expression, and promoter activity. To further ensure that TNF-α-induced cPLA_2_ expression was mediated via p42/p44 MAPK, as shown in Fig. 3C, transfection with p42 siRNA significantly down-regulated p42 protein expression and subsequently led to a decrease of cPLA_2_ protein expression by TNF-α. Finally, we showed that TNF-α stimulated p42/p44 MAPK phosphorylation in a time-dependent manner, which was reduced by PD98059 during the period of observation (Fig. 3D). These data indicated that MEK1/2-p42/p44 MAPK cascade was involved in TNF-α-induced cPLA_2_ expression in HPAEpiCs.

**Figure 3:** p42/p44 MAPK is involved in TNF-α-induced cPLA_2_ expression. (A) Cells were pretreated with PD98059 for 1 h, and then incubated with TNF-α for 24 h. The protein levels of cPLA_2_ were determined by Western blot. (B) Cells were pretreated with PD98059 (10 µM) for 1 h, and then incubated with TNF-α for 6 h. cPLA_2_ mRNA levels and promoter activity were determined. (C) Cells were transfected with scrambled or p42 siRNA, and then incubated with TNF-α for 24 h. The protein levels of p42 and cPLA_2_ were determined. (D) Cells were pretreated with or without PD98059 (10 µM) for 1 h, and then incubated with TNF-α for the indicated time intervals. The levels of phospho-p42/p44 MAPK were determined. Data are expressed as mean±S.E.M. of three independent experiments. *P<0.05; ^#^ *P*<0.01, as compared with the cells exposed to TNF-α alone.

### TNF-α induces cPLA_2_ expression via p38 MAPK in HPAEpiCs

cPLA_2_ expression induced by LPS has been shown to be mediated through p38 MAPK in canine airway smooth muscle cells [19]. To determine whether p38 MAPK was also involved in TNF-α-induced cPLA_2_ expression in HPAEpiCs, a p38 MAPK inhibitor, SB202190 was used. As shown in Figs. 4A and B, pretreatment with SB202190 inhibited TNF-α-induced cPLA_2_ protein and mRNA expression, and promoter activity. To further ensure that TNF-α-induced cPLA_2_ expression was mediated via p38 MAPK in these cells, as shown in Fig. 4C, transfection with p38 siRNA significantly down-regulated p38 MAPK protein expression and subsequently led to a decrease of cPLA_2_ protein expression by TNF-α. Finally, we showed that TNF-α stimulated p38 MAPK phosphorylation in a time-dependent manner, which was reduced by SB202190 during the period of observation (Fig. 4D). These data indicated that p38 MAPK cascade was involved in TNF-α-induced cPLA_2_ expression in HPAEpiCs.

RETRACTED

**Figure 4:** p38 MAPK is involved in TNF-α-induced cPLA_2_ expression. (A) Cells were pretreated with SB202190 for 1 h, and then incubated with TNF-α for 24 h. The protein levels of cPLA_2_ were determined by Western blot. (B) Cells were pretreated with SB202190 (10 µM) for 1 h, and then incubated with TNF-α for 6 h. cPLA_2_ mRNA levels and promoter activity were determined. (C) Cells were transfected with scrambled or p38 siRNA, and then incubated with TNF-α for 24 h. The protein levels of p38 and cPLA_2_ were determined. (D) Cells were pretreated with or without SB202190 (10 µM) for 1 h, and then incubated with TNF-α for the indicated time intervals. The levels of phospho-p38 MAPK were determined. Data are expressed as mean±S.E.M. of three independent experiments. ^#^ *P*<0.01, as compared with the cells exposed to TNF-α alone.

### TNF-α enhances cPLA_2_ expression via JNK1/2 in HPAEpiCs

Expression of cPLA_2_ in lung epithelial cells and non-small cell lung cancer is mediated by Sp1 and c-Jun through JNK1/2 activation [30]. To characterize the role of JNK1/2 in TNF-α-induced cPLA_2_ expression in HPAEpiCs, a selective inhibitor of JNK1/2, SP600125, was used. As shown in Figs. 5A and B, pretreatment with SP600125 blocked TNF-α-induced cPLA_2_ protein and mRNA expression, and promoter activity. To further ensure that TNF-α-induced cPLA_2_ expression was mediated via JNK1/2 in HPAEpiCs, as shown in Fig. 5C, transfection with JNK2 siRNA significantly down-regulated JNK2 expression and subsequently led to a decrease of cPLA_2_ protein expression in response to TNF-α. Finally, we showed that TNF-α stimulated JNK1/2 phosphorylation in a time-dependent manner, which was reduced by SP600125 during the period of observation (Fig. 5D). These results suggested that JNK1/2 activation was required for TNF-α-induced cPLA_2_ expression in HPAEpiCs.

RETRACTED

**Figure 5:** JNK1/2 is involved in TNF-α-induced cPLA_2_ expression. (A) Cells were pretreated with SP600125 for 1 h, and then incubated with TNF-α for 24 h. The protein levels of cPLA_2_ were determined by Western blot. (B) Cells were pretreated with SP600125 (10 µM) for 1 h, and then incubated with TNF-α for 6 h. cPLA_2_ mRNA levels and promoter activity were determined. (C) Cells were transfected with scrambled or JNK2 siRNA, and then incubated with TNF-α for 24 h. The protein levels of JNK2 and cPLA_2_ were determined. (D) Cells were pretreated with or without SP600125 (10 µM) for 1 h, and then incubated with TNF-α for the indicated time intervals. The levels of phospho-JNK1/2 were determined. Data are expressed as mean±S.E.M. of three independent experiments. ^#^ *P*<0.01, as compared with the cells exposed to TNF-α alone.

### AP-1 is involved in TNF-α-induced cPLA_2_ expression and PGE_2_ release in HPAEpiCs

AP-1 is a transcription factor which is a heterodimeric protein composed of proteins belonging to the c-Fos, c-Jun, ATF, and JDP families [21], which regulates gene expression induced by various stimuli, including cytokines, growth factors, stress, and bacterial and viral infections [21]. To characterize the role of AP-1 in TNF-α-induced cPLA_2_ expression in HPAEpiCs, a selective inhibitor of AP-1, Tanshinone IIA, was used. As shown in Figs. 6A and B, pretreatment with Tanshinone IIA blocked TNF-α-induced cPLA_2_ protein and mRNA expression, and promoter activity. To further ensure that TNF-α-induced cPLA_2_ expression was mediated via AP-1 in HPAEpiCs, as shown in Fig. 6C, transfection with c-Jun or c-Fos siRNA significantly down-regulated c-Jun or c-Fos expression and subsequently led to a decrease of cPLA_2_ protein expression by TNF-α. To further confirm the role of AP-1 in TNF-α-mediated cPLA_2_ promoter induction, point-mutated AP-1 cPLA_2_ promoter construct was used. As shown in Fig. 6D, TNF-α-stimulated cPLA_2_ promoter activity was prominently lost in HPAEpiCs transfected with point-mutated AP-1 cPLA_2_ promoter. Finally, we found that pretreatment with PD98059, SB202190, SP600125, or Tanshinone IIA markedly reduced TNF-α-induced PGE_2_ release in these cells (Fig. 6E). Thus, these data suggested that TNF-α induces cPLA_2_ expression via an AP-1 signaling in HPAEpiCs.

**Figure 6:** AP-1 is involved in TNF-α-induced cPLA_2_ expression. (A) Cells were pretreated with Tanshinone IIA (TSIIA) for 1 h, and then incubated with TNF-α for 24 h. The protein levels of cPLA_2_ were determined by Western blot. (B) Cells were pretreated with Tanshinone IIA (TSIIA), and then incubated with TNF-α for 6 h. cPLA_2_ mRNA levels and promoter activity were determined. (C) Cells were transfected with scrambled, c-Jun, or c-Fos siRNA, and then incubated with TNF-α for 24 h. The protein levels of c-Jun, c-Fos, and cPLA_2_ were determined. (D) Cells were transfected with pGL3-empty, wild-type cPLA_2_ promoter, or AP-1-mutated cPLA_2_ promoter, and then incubated with TNF-α for 6 h. The promoter activity of cPLA_2_ was determined in the cell lysates. (E) Cells were pretreated with PD98059 (10 µM), SB202190 (10 µM), SP600125 (10 µM), or Tanshinone IIA (TSIIA; 10 µM) for 1 h, and then incubated with TNF-α for 24 h. The media were collected and analyzed for PGE_2_ release. Data are expressed as mean±S.E.M. of three independent experiments. ^#^ *P*<0.01, as compared with the cells exposed to TNF-α alone (A, B, and E). ^#^ *P*<0.01, as compared with cells transfected with wild-type cPLA_2_ promoter stimulated by TNF-α (D).

RETRACTED

### TNF-α stimulates p300/ATF2/c-Jun/c-Fos complex formation in HPAEpiCs

ATF2 is a member of the ATF/cyclic AMP-responsive element binding protein family of transcription factors and implicated in inflammatory responses [31]. To ensure that TNF-α-induced cPLA_2_ expression was mediated via ATF2 in HPAEpiCs, as shown in Fig. 7A, transfection with ATF2 siRNA significantly down-regulated ATF2 expression and subsequently led to a decrease of cPLA_2_ protein expression by TNF-α. On the other hand, we demonstrated that TNF-α time-dependently induced c-Fos and c-Jun protein expression or c-Jun and ATF2 phosphorylation in these cells (Fig. 7B). We further investigated the relationship between MAPKs and AP-1 in TNF-α-stimulated HPAEpiCs. As shown in Fig. 7C, TNF-α-enhanced ATF2 phosphorylation was inhibited by SB202190, but not PD98059 and SP600125. However, c-Jun phosphorylation stimulated by TNF-α was inhibited by SP600125, but not PD98059 oand SB202190. Thus, we suggested that TNF-α-induced cPLA_2_ expression is mediated through AP-1 activation which is regulated by p38 MAPK and JNK1/2 but not p42/p44 MAPK in HPAEpiCs.

**Figure 7:** TNF-α stimulates p300/ATF2/c-Jun/c-Fos complex formation. (A) Cells were transfected with scrambled or ATF2 siRNA, and then incubated with TNF-α for 24 h. The protein levels of ATF2 and cPLA_2_ were determined. (B) Cells were incubated with TNF-α for the indicated time intervals. The levels of c-Fos, c-Jun, phospho-c-Jun, and phospho-ATF2 were determined. (C) Cells were pretreated with PD98059, SB202190, or SP600125, and then incubated with TNF-α for 90 min or 15 min. The levels of phospho-ATF2 and phospho-c-Jun were determined. (D) Cells were incubated with TNF-α for the indicated time intervals. The cell lysates were subjected to immunoprecipitation using an anti-p300 antibody, and then the immunoprecipitates were analyzed by Western blot using an anti-c-Fos, anti-c-Jun, anti-ATF2, or anti-p300 antibody. (E) Cells were treated with TNF-α for the indicated time intervals, and then ChIP assay was performed. Chromatin was immunoprecipitated using an anti-p300, anti-ATF2, anti-c-Fos, or anti-c-Jun antibody. One percent of the precipitated chromatin was assayed to verify equal loading (Input). Data are expressed as mean±S.E.M. of three independent experiments. ^#^ *P*<0.01, as compared with the cells exposed to TNF-α alone.

RETRACTED

The transcriptional co-activator p300 displays an intrinsic HAT activity which participates in transcriptional activation through the destabilization of nucleosome structure. p300 is involved in the activity of several transcription factors that are nuclear endpoints of intracellular signal transduction pathways [20]. Moreover, co-immunoprecipitation study revealed that TNF-α-stimulated p300 directly associated with c-Fos, c-Jun, or ATF2 in a time-dependent manner with a maximal response within 30 min. Finally, the *in vivo* recruitment of p300, ATF2, c-Fos, and c-Jun to the cPLA_2_ promoter was assessed by a ChIP assay. *In vivo* binding of p300, ATF2, c-Fos, and c-Jun to the cPLA_2_ promoter occurred as early as 15 min and was sustained for 30 min following TNF-α stimulation (Fig. 7E).

### TNF-α induces leukocyte accumulation in BAL and cPLA_2_ mRNA expression in mice via MAPKs and AP-1

TNF-α has been shown to induce ROS generation via NADPH oxidase activation, which in turn initiates the activation of various signaling pathways, including PKCs, PI3K/Akt, and MAPKs or transcription factors, such as NF-κB and AP-1, and ultimately induces expression of cPLA_2_. Moreover, cPLA_2_ induction may trigger airway and pulmonary diseases, such as asthma and COPD [1]. To further confirm the effects of TNF-α on animal models, mice were (i.p.) injected with PD98059, SB202190, SP600125, or Tanshinone IIA, and then administrated by oropharyngeal route with TNF-α for 24 h. As shown in Fig. 8A, TNF-α markedly induced cPLA_2_ mRNA expression in lung tissues of mice, which was reduced by PD98059, SB202190, SP600125, or Tanshinone IIA. In addition, we also showed that PD98059, SB202190, SP600125, Tanshinone IIA, or AACOCF_3_ (an inhibitor of cPLA_2_) reduced TNF-α-induced leukocyte count in BAL fluid of mice (Fig. 8B). PGE_2_, one of the major PGs products, exerts its biological activities by binding to specific cell surface receptors, designated PGE_2_ receptors (EPs). To investigate whether PGE_2_ could induce leukocyte count in BAL fluid of mice, AH 6809 (an EP1 and EP2 receptor antagonist), SC-19220 (an EP1 receptor antagonist), or GW627368X (an EP4 receptor antagonist) was used. As shown in Fig. 8C, these three EP receptor antagonists reduced TNF-α-induced leukocyte count in BAL fluid of mice. These data suggested that TNF-α may promote leukocyte accumulation and lung inflammation via cPLA_2_-mediated PGE_2_ release to cause airway and pulmonary diseases, such as asthma and COPD.

RETRACTED

**Figure 8:** TNF-α induces leukocyte accumulation in BAL and cPLA_2_ mRNA expression in mice via MAPKs and AP-1. (A) Mice were i.p. given one dose of PD98059, SB202190, SP600125, or Tanshinone IIA (2 mg/kg) for 1 h before TNF-α treatment, and sacrificed after 24 h. Lung tissues were homogenized to extract mRNA. The levels of cPLA_2_ mRNA were determined by real-time PCR. (B, C) Mice were i.p. given one dose of PD98059, SB202190, SP600125, Tanshinone IIA, AACOCF_3_, AH 6809, SC-19220, or GW627368X (2 mg/kg) for 1 h before TNF-α treatment, and sacrificed after 24 h. BAL fluid was acquired and leukocyte count was determined by a hemocytometer. (D) Schematic representation of the signaling pathways involved in the TNF-α-induced cPLA_2_ expression in HPAEpiCs. TNF-α-induced cPLA_2_ expression and PGE_2_ release are mediated through p38 MAPK- and JNK1/2-dependent p300/c-Fos/c-Jun/ATF2 complex formation in HPAEpiCs.

## Discussion

Asthma and COPD are pulmonary disorders characterized by various degrees of inflammation and tissue remodeling. Up-regulation of cPLA_2_ expression by mesenchymal cells in several extra-pulmonary sites may play a key role in generation of PGE_2_, known as a biologically active lipid mediator implicated in inflammatory responses [32]. TNF-α has been confirmed to induce the late-phase airway hyperresponsiveness and inflammation mediated through activation of cPLA_2_ [33], but little is known about the intracellular signaling pathways leading to its expression. TNF-α has also been shown to activate MAPKs pathways in several cell types [18], [34]. In addition, AP-1 activity is regulated by multiple mechanisms, including phosphorylation by various MAPKs [22]. Among MAPKs, JNK1/2 predominantly plays an important role in TNF-α-induced AP-1 activity, which contributes to the induction of TNF-α-targeted genes [23]. However, in HPAEpiCs, whether TNF-α-induced cPLA_2_ expression was mediated through the activation of MAPKs and AP-1 was still unknown. In this study, TNF-α induced cPLA_2_ expression and PGE_2_ production which were attenuated by pretreatment with the inhibitors of MEK1/2 (PD98059), p38 MAPK (SB202190), JNK1/2 (SP600125), and AP-1 (Tanshinone IIA) or transfection with siRNAs of p42, p38, JNK2, c-Fos, c-Jun, ATF2, and TNFR1. Here, our results suggested that in HPAEpiCs, TNF-α-induced cPLA_2_ expression associated with PGE_2_ release was, at least in part, mediated through JNK1/2- and p38 MAPK-dependent p300-AP-1 signaling pathway. These results demonstrated that MAPKs and AP-1 may be the critical components implicated in cPLA_2_ expression and PGE_2_ synthesis in TNF-α-challenged HPAEpiCs.

RETRACTED

Accumulating evidence demonstrates that TNF-α may activate downstream protein kinases leading to the expression of inflammatory proteins [18], [29]. All known responses to TNF-α are triggered by binding to one of two distinct receptors, designated as TNFR1 and TNFR2 [29]. However, based on cell culture experiments and studies with receptor knockout mice, both the proinflammatory and the programmed cell death pathways that are activated by TNF-α, and associated with tissue injury, are largely mediated through TNFR1 [29], [35]. In contrast, TNFR2 has been shown to mediate signals that promote tissue repair and angiogenesis [36]. Indeed, in HPAEpiCs, we also showed that TNFR1 plays a key role in mediating TNF-α-induced inflammatory responses.

Several extracellular stimuli elicit a broad spectrum of biological responses mediated through activation of MAPKs, including p42/p44 MAPK, p38 MAPK, and JNK1/2. Since TNF-α plays an important role in different cellular responses, the activation of these MAPKs is not necessarily restricted to TNF-α-induced cPLA_2_ expression. For example, activation of JNK1/2 and p42/p44 MAPK is required for up-regulation of cPLA_2_ in response to oncogenic Ras in normal epithelial cells [16]. In canine airway smooth muscle cells, up-regulation of cPLA_2_ by LPS is mediated through these MAPKs pathways [19]. Moreover, IL-1β induces expression of cPLA_2_ in human airway smooth muscle cells, which is regulated by p38 MAPK and JNK1/2, but not p42/p44 MAPK [37]. In the present study, our results demonstrated that activation of p42/p44 MAPK, p38 MAPK, or JNK1/2 was necessary for TNF-α-induced cPLA_2_ expression and PGE_2_ release in HPAEpiCs. These results were consistent with the reports indicating that activation of MAPKs plays a pivotal role in the expression of cPLA_2_ in various cell types [19], [20].

AP-1 is a dimeric transcription factor comprising proteins from several families whose common denominator is the possession of basic leucine zipper (bZIP) domains that are essential for dimerization and DNA binding. It has been well established that inflammatory responses following exposure to extracellular stimuli are highly dependent on activation of AP-1 which plays an important role in the expression of several target genes [22]. Our group has indicated that IL-1β could induce cPLA_2_ expression via p42/p44 MAPK- and JNK1/2-dependent AP-1 activation in RA synovial fibroblasts (RASFs) [38]. In addition, we also demonstrated that cigarette smoke extract (CSE) induces cPLA_2_ expression via MAPKs, AP-1, and NF-κB in human tracheal smooth muscle cells [39]. Here, in HPAEpiCs, we also found that TNF-α-induced cPLA_2_ expression and PGE_2_ release was decreased via AP-1 inhibition. On the other hand, we also demonstrated that TNF-α could enhance c-Jun and c-Fos protein expression, which may promote TNF-α-mediated induction of inflammatory genes. The transcriptional activity of c-Jun is regulated by phosphorylation at Ser^63^ and Ser^73^ through JNK1/2 [22]. The transcription factor ATF2 (also called CRE-BP1) binds to both AP-1 and CRE DNA response elements and is a member of the ATF/CREB family of leucine zipper proteins. Various forms of cellular stresses, including genotoxic agents, inflammatory cytokines, and UV irradiation, stimulate the transcriptional activity of ATF2. Cellular stresses activate ATF2 by phosphorylation of Thr^69^ and Thr^71^ [21], [22]. Moreover, in HPAEpiCs, TNF-α could stimulate c-Jun and ATF2 phosphorylation in a time-dependent manner. We further established that p38 MAPK, but not p42/p44 MAPK and JNK1/2 plays a key role in mediating TNF-α-induced ATF2 activation in these cells. However, TNF-α-induced c-Jun phosphorylation was regulated via JNK1/2 activation. Although p42/p44 MAPK was involved in TNF-α-induced cPLA_2_ expression, which was not mediated through activation of ATF2 and c-Jun in HPAEpiCs. In the future, we will investigate whether p42/p44 MAPK may regulate other transcription factors, such as NF-κB or Elk-1, leading to cPLA_2_ expression.

RETRACTED

In non-small cell lung cancer cells, cPLA_2_ gene expression can be regulated by various transcription factors, including Sp1 and c-Jun [30]. Both Sp1 and c-Jun have been reported to interact with co-activator, p300, one of HAT members [40], [41]. HATs, such as p300 and CREB binding protein (CBP) act as protein bridges, thereby connecting different transcriptional activators via protein-protein interactions to the basal transcriptional machinery, including transcription factor IIB (TFIIB), TATA-binding protein, and the RNA polymerase II complex [42]. They also function as a scaffolding protein which builds a multi-component transcriptional regulatory complex. Raised activity of intrinsic HAT may cause remodeling of chromatin structure by acetylation of the NH_2_ terminus of core nucleosomal histones [42]. Chromatin remodeling after p300/CBP associated with histone acetylation is believed to participate in active transcription of pro-inflammatory genes upon stimulation by various mediators. Here, we found that TNF-α time-dependently induced p300/c-Fos/c-Jun/ATF2 complex formation in HPAEpiCs. Finally, we also established that TNF-α markedly induced *in vivo* binding of p300, ATF2, c-Fos, and c-Jun to the cPLA_2_ promoter.

Based on the observation from literatures and our findings, Fig. 8D reveals a model for the signaling mechanisms implicated in TNF-α-induced cPLA_2_ expression and PGE_2_ release in HPAEpiCs. Indeed, previous study showed that cigarette smoke extract (CSE) induced cPLA_2_ expression in airway smooth muscle cells via the NADPH oxidase-dependent p42/p44 MAPK and p38 MAPK/c-Fos and JNK1/2/c-Jun/p300 pathways [39]. In addition, our group also indicated that TNF-α induced cPLA_2_ expression through MAPKs, and then the activated MAPKs regulated the activity of p300 and acetylation of histone H4 and hence led to cPLA_2_ expression [20]. Chi et al. demonstrated that IL-1β induced cPLA_2_ expression via activation of p42/p44 MAPK and JNK1/2, which further stimulated AP-1 activation in rheumatoid arthritis synovial fibroblasts [38]. However, this study is the first to demonstrate that in HPAEpiCs, the mechanisms underlying TNF-α-mediated activation of MAPKs and AP-1 was required for the expression of cPLA_2_. Finally, association of p300, ATF2, c-Jun, and c-Fos led to cPLA_2_ gene transcription. The mechanisms by which TNF-α induced cPLA_2_ expression may be an important link in the pathogenesis of lung inflammatory diseases. Therefore, understanding the mechanisms underlying TNF-α-induced cPLA_2_ expression in HPAEpiCs is important to develop new therapeutic strategies.
